The article "The Efficacy of Targeted Perioperative Management for Diabetic Patients with Traumatic Calcaneal Fractures" was retracted in 2023. Reasons: unreliable results or conclusions; concerns about the data; concerns about the results or conclusions; concerns about the peer review.

# The Efficacy of Targeted Perioperative Management for Diabetic Patients with Traumatic Calcaneal Fractures

**DOI:** 10.1155/2022/1294416

**Published:** 2022-06-28

**Authors:** Sibin Hao, Yunpeng Liu, Mingtai Yu, Fang Sun, Dezhang Wang

**Affiliations:** Department of Hand and Foot Surgery, Jinan Zhangqiu District People's Hospital, Jinan, China

## Abstract

**Objective:**

To assess the efficacy of targeted perioperative management for diabetic patients with traumatic calcaneal fractures.

**Methods:**

Between April 2020 and December 2020, 100 diabetic patients with traumatic calcaneal fractures treated in our institution satisfying the inclusion criteria were enrolled and assigned to receive either conventional treatment with surgery or plaster fixation (observation group) or targeted treatment with surgery or plaster fixation (experimental group) via the random number table method, with 50 patients in each group. All eligible patients were followed up for 1 year postoperatively. Outcome measures included length of hospital stay, recovery time, fracture healing, duration of postoperative wound drainage, complication rate, blood glucose, and treatment satisfaction. The Maryland score was used for the assessment of foot function.

**Results:**

The duration of postoperative wound drainage, length of hospital stay, and recovery time in the experimental group (3.63 ± 1.04 d, 12.13 ± 3.77 d, and 111.22 ± 16.24 d) were significantly shorter than those in the observation group (5.71 ± 2.34 d, 15.28 ± 4.42 d, 123.10 ± 22.82 d) (*P* < 0.01). The experimental group obtained a markedly higher complete healing rate versus the observation group (*P* < 0.001). A significantly lower complication rate was observed in the experimental group than in the observation group (*P* < 0.05). The Maryland scores results were dichotomized into good (≥75 points) and poor (<75 points). The experimental group showed significantly higher Maryland scores good rate and treatment satisfaction versus the observation group (*P* < 0.01). The experimental group patients were associated with better postoperative fasting glucose and 2 h postprandial glucose versus those in the observation group (*P* < 0.05).

**Conclusion:**

Targeted treatment in the perioperative management of diabetic patients with traumatic calcaneal fractures significantly promotes the recovery of patients, reduces the incidence of complications, increases treatment satisfaction, and ameliorates the doctor-patient relationship.

## 1. Introduction

The calcaneus is the largest tarsal bone in the human body and is an important component of the foot arch. The calcaneus has a complex anatomy and irregular morphology, with six surfaces and four articular facets. The calcaneus is the common posterior jaw of the posterior branch of the medial and lateral longitudinal arches of the foot, and its anterior end supports the talus and bears the weight of the body. The upper part of the calcaneus consists of three articular surfaces, which, together with the talus, comprise the subtalar joint complex and maintain the mechanical stability of the subtalar joint. The posterior articular surface of the calcaneus bears the majority of the body mass. Calcaneal fractures are a common clinical fracture type and are associated with up to 60% of tarsal fractures. Treatment of calcaneal fractures is complicated and prone to various complications, so how to ensure effective treatment outcomes and lower the incidence of complications remains one of the pressing issues to be addressed in orthopedics. Surgery is the mainstay of treatment for poor alignment of broken bones, and cast fixation is adopted for good alignment. Diabetes mellitus is a common metabolic disorder with a high prevalence worldwide. It is characterized by hyperglycemia elicited by defective insulin secretion, insulin action, or both. Statistics showed that the proportion of diabetic patients worldwide was approximately 25.6% in 2015. The disease is highly liable to complications, such as cardiovascular and cerebrovascular diseases, neurological diseases, and nephropathies, and may lead to malignant neoplastic diseases in the event of disease deterioration without timely treatment. Diabetes is a major risk factor for cardiovascular disease. The treatment of diabetes is complicated and no significant breakthroughs have been achieved. Thus, early screening and diagnosis are of great significance. The high blood glucose of diabetic patients with traumatic calcaneal fractures may retard fracture healing, and the patients are predisposed to postoperative complications such as incisional infections, which compromise the recovery of foot function and the quality of life of the patients [1–3]. It has been suggested that the combination of perioperative targeted therapeutic interventions contributes to reducing postoperative complications and shortening the recovery time [4, 5]. To this end, this study was conducted to assess the efficacy of targeted treatment in the perioperative management of diabetic patients with traumatic calcaneal fractures.

The article "The Efficacy of Targeted Perioperative Management for Diabetic Patients with Traumatic Calcaneal Fractures" was retracted in 2023. Reasons: unreliable results or conclusions; concerns about the data; concerns about the results or conclusions; concerns about the peer review.

## 2. Materials and Method

### 2.1. Baseline Data

Between April 2020 and December 2020, 100 patients with traumatic calcaneal fractures combined with diabetes mellitus treated in our institution satisfying the inclusion criteria were enrolled and assigned to receive either conventional treatment with surgery or plaster fixation (observation group) or targeted treatment with surgery or plaster fixation (experimental group) via random number table methods, with 50 patients in each group. In the observation group, there were 24 females and 26 males, aged between 25 and 66 years, with an average age of 38.5 ± 4.2 years. In terms of the cause of injury, there were 21 cases of traffic accidents, 17 cases of falling from height, and 12 cases of sports injuries; in terms of Sanders fracture classification, there were 17 cases of type II, 21 cases of type III, and 12 cases of type IV. In the experimental group, there were 23 females and 27 males, aged between 24 and 66 years, with a mean age of (38.3 ± 4.4) years. In terms of the cause of injury, there were 22 cases of traffic accidents, 16 cases of falling from height, and 12 cases of sports injuries; in terms of Sanders fracture classification, there were 19 cases of type II, 20 cases of type III, and 11 cases of type IV. The studies involving human participants were reviewed and approved by the Ethics Committee of Jinan Zhangqiu District People's Hospital (Approval no. 97770/93).

Inclusion criteria were as follows: patients with calcaneal fractures confirmed by imaging and who met the indications for surgical treatment; patients who were diagnosed with diabetes mellitus with fasting blood glucose of ≥7.0 mmol/L and 2 h postprandial blood glucose (2hPBG) of ≥11.1 mmol/L; and patients who voluntarily participated in the study and provided written informed consent were included.

Exclusion criteria were as follows: patients with minor fractures, not requiring inpatient surgery; patients with cardiovascular, cerebrovascular, endocrine, liver, and kidney insufficiency, and other chronic medical diseases; and patients with the withdrawal of consent were considered ineligible and excluded.

There was no statistically significant difference between the two groups in terms of baseline features such as gender, age, cause of injury, fasting glucose, and fracture types (*P* > 0.05) (Table 1). The study was approved by the medical ethics review board.

### 2.2. Methods

Patients in the observation group received conventional treatment, including precautions, health education, postoperative basic maintenance, and discharge instructions. Patients in the experimental group received targeted treatment, including preoperative, intraoperative, and postoperative management [6, 7].

#### 2.2.1. Preoperative Management

(1) The nursing staff actively communicated with the patients to understand their psychological state and helped them relieve negative emotions to improve their treatment cooperation [8, 9]. (2) The patients were given health education, including the causes of diabetes mellitus, blood glucose control, and care for calcaneal fractures. Patients were also given dietary instructions for strict control of sugar intake and were advised to have more coarse grains, vegetables, fruits, high protein, and high calcium foods to promote recovery [10].

The article "The Efficacy of Targeted Perioperative Management for Diabetic Patients with Traumatic Calcaneal Fractures" was retracted in 2023. Reasons: unreliable results or conclusions; concerns about the data; concerns about the results or conclusions; concerns about the peer review.

#### 2.2.2. Intraoperative Management

(1) Patients who required surgery were treated with incisional repositioning and internal fixation. An enlarged L-shaped incision was used, and a suitable lateral heel plate and screws were used for fixation after satisfactory repositioning. The closure of the surgical incision was performed by the same operator and assistant, and the subcutaneous tissues were closed intermittently to avoid dead cavities, followed by the placement of a drainage tube. Disposable skin sutures (Changzhou Heraeus PWHW35) were applied to staple the incision. (2) Patients who did not need surgery were treated with plaster fixation.

#### 2.2.3. Postoperative Management

(1) After the procedure, the patient was maintained in a prone position and the affected limb was elevated to an appropriate angle to facilitate venous blood return. The blood circulation, skin color, and temperature of the patient's foot were monitored, and antibiotics were administered to prevent infection [11, 12]. The patients received insulin injections and their blood glucose was determined thrice daily for the adjustment of their insulin dose. (2) The patients' wounds were monitored, and the property and color of the drains were observed in case of abnormalities. The drainage tubes were removed 3 d after the surgery. The affected limbs were checked for swelling, and the patients were instructed to perform ankle exercises. If necessary, the affected limbs were massaged to promote blood circulation. Exercise instruction was given based on recovery. (3) Diabetic patients with high levels of D-dimer expression are prone to lower limb deep vein thrombosis, so drugs to dilate blood vessels and improve peripheral blood circulation were administered before and after surgery to prevent limb deep vein thrombosis. The patients were instructed to perform active exercises such as ankle exercises and quadriceps, and their family members were guided to massage the affected limb of the patients from the distal end to the proximal end. Lower extremity vascular ultrasound was performed to clarify the disease condition if the affected extremity was severely swollen, and early symptoms of pulmonary embolism were managed promptly.

#### 2.2.4. Blood Glucose Management

After understanding the patient's living habits and diet structure, a tailored diet protocol was formulated to control the patient's daily intake of sugar, fat, and protein for effective glucose and blood lipid management. Patients with traumatic fractures and diabetes mellitus suffer severe physical and mental shock, resulting in massive physical exertion, negative nitrogen balance, increased secretion of endocrine hormones, and elevated blood glucose. The patients were instructed to eat nutritious and low-sugar foods, with whole wheat flour in place of refined flour and mixed grain rice in place of white rice. Patients were advised to consume more vegetables and proteins such as milk, lean meat, poultry, eggs, fish, and soy products. Patients were advised against greasy foods such as peanuts and nuts. They were also instructed to have a daylong stream of mini-meals and increase consumption of calcium-containing foods.

The article "The Efficacy of Targeted Perioperative Management for Diabetic Patients with Traumatic Calcaneal Fractures" was retracted in 2023. Reasons: unreliable results or conclusions; concerns about the data; concerns about the results or conclusions; concerns about the peer review.

### 2.3. Outcomes

The hospital-made questionnaire and pathology records were used to compare the length of hospital stay, recovery time, fracture healing, duration of postoperative wound drainage, complication rate, blood glucose changes, and treatment satisfaction between the two groups, and the Maryland score was used to assess the patients' foot function.

1. *Criteria for Fracture Healing*. Complete healing: there were no tenderness and no percussion pain along the longitudinal axis of the limb, and no discomfort from self-elevation of the affected limb, and the fracture line disappeared on X-ray. Basic healing: there were no tenderness and no percussion pain along the longitudinal axis of the limb, with possible discomfort from self-elevation of the affected limb, and the fracture line was blurred on X-ray.
2. *Complications.* The complications during treatment include surgical wound infection, delayed healing, healing deformity, and joint pain.
3. *Determination of Blood Glucose.* 4 mL of peripheral venous blood was collected from all eligible patients before and after treatment, and the serum was isolated by centrifugation at 3000 r/min for 15 min (centrifugal radius of 10 cm) using a C1012-E blood centrifuge (Wuxi Microchromatography Biotechnology Co. Ltd.) with original reagents to determine serum fasting blood glucose and postprandial 2 h blood glucose level.
4. *Treatment Satisfaction*. A questionnaire prepared by our hospital was used, with a total of 16 questions. The total score is 48 points, with 3 points for satisfied, 2 points for basic satisfied, and 0 points for dissatisfied. The formula for score calculation is as follows: the sum of the scores obtained from the questionnaire/48 *∗* 100%. Satisfied: final score >40 points; basically satisfied: final score of 24–40 points; unsatisfied: final score ≤24 points.
5. *Maryland Scoring Criteria*. 40 points: no obvious pain; 30 points: occasional mild pain; 20 points: occasional moderate pain; 0 points: frequent severe pain. 10 points: no restriction of activity; 8 points: slight restriction of activity, 0 points: severe restriction of activity. 10 points: normal healing; 8 points: slight deformity; 6 points: moderate deformity; 0 points: severe deformity. The score was 100 points, in which excellent was ≥90 points, good was 75–90 points, moderate was 50–74 points, and poor was ≤50 points.

The article "The Efficacy of Targeted Perioperative Management for Diabetic Patients with Traumatic Calcaneal Fractures" was retracted in 2023. Reasons: unreliable results or conclusions; concerns about the data; concerns about the results or conclusions; concerns about the peer review.

### 2.4. Statistical Analysis

SPSS 20.0 was used for data analysis, and GraphPad Prism 8 was used to plot the graphics. The measurement data are expressed as mean ± standard deviation and analyzed using the independent samples *t*-test. The count data are expressed as cases (%) and analyzed using the chi-square test. Hierarchical data were compared using the rank-sum test. Differences were considered statistically significant at *P* < 0.05.

## 3. Results

### 3.1. Length of Hospital Stay and Recovery Time

The length of hospital stay was (12.13 ± 3.77) d and (15.28 ± 4.42) d, the recovery time was (111.22 ± 16.24) d and (123.10 ± 22.82) d, and the duration of postoperative wound drainage was (3.63 ± 1.04) d and (5.71 ± 2.34) d in the experimental group and the observation group, respectively. A significantly shorter length of hospital stay, recovery time, and duration of postoperative wound drainage were observed in the experimental group versus the observation group (*P* < 0.01) (Table 2).

### 3.2. Complete Fracture Healing Rate

All patients in the experimental group showed complete healing, with a healing rate of 100%. The observation group had 33 cases of complete healing and 17 cases of basic healing, with a healing rate of 66% (*X*^2^ = 20.482, *P* < 0.001) (Figure 1).

### 3.3. Comparison of Complication Rates

The experimental group showed 1 case of wound infection, 0 cases of delayed healing, 1 case of healing deformity, and 0 cases of joint pain, with a complication rate of 4% (2 cases). The observation group showed 3 cases of wound infection, 1 case of delayed healing, 2 cases of healing deformity, and 3 cases of joint pain, with a complication rate of 18% (9 cases). The experimental group had significantly lower complication rates than those of the observation group (*X*^2^ = 5.005, *P*=0.025) (Table 3).

### 3.4. Maryland Scores

The experimental group had 35 cases of excellent, 11 cases of good, 4 cases of moderate, and 0 cases of poor, with a good rate of 92% (46 cases). The observation group had 11 cases of excellent, 21 cases of good, 11 cases of moderate, and 7 cases of poor, with a good rate of 64% (32 cases). The experimental group showed a higher good rate than the observation group (*X*^2^ = 22.844, *P* < 0.001) (Figure 2).

The article "The Efficacy of Targeted Perioperative Management for Diabetic Patients with Traumatic Calcaneal Fractures" was retracted in 2023. Reasons: unreliable results or conclusions; concerns about the data; concerns about the results or conclusions; concerns about the peer review.

### 3.5. Comparison of Treatment Satisfaction

The experimental group had 37 cases of satisfied, 11 cases of basically satisfied, and 2 cases of dissatisfied, with a total satisfaction rate of 96% (48/50). The observation group had 20 cases of satisfied, 13 cases of basically satisfied, and 17 cases of dissatisfied, with a total satisfaction rate of 66% (33). Treatment satisfaction was significantly higher in the experimental group than in the observation group (*X*^2^ = 14.620, *P* < 0.01) (Table 4).

### 3.6. Comparison of Blood Glucose

In the experimental group, the pretreatment fasting blood glucose level was (8.33 ± 1.13) mmol/L, the posttreatment fasting blood glucose level was (7.01 ± 2.03) mmol/L, the pretreatment 2 h postprandial blood glucose level was (15.28 ± 2.35) mmol/L, and the posttreatment 2 h postprandial blood glucose level was (12.38 ± 2.21) mmol/L. In the observation group, the pretreatment fasting blood glucose level was (8.42 ± 1.22), the posttreatment fasting blood glucose level was (7.96 ± 1.99) mmol/L, the pretreatment 2 h postprandial blood glucose level was (15.36 ± 2.42) mmol/L, and the posttreatment 2 h postprandial blood glucose level was (14.22 ± 2.16) mmol/L. The experimental group showed better blood glucose levels than the observation group (*P*=0.02 or <0.001) (Table 5).

## 4. Discussion

Fluctuation of blood glucose in diabetic patients may be attributed to intraoperative stress. Thus, patients' blood glucose during perioperative management requires timely control and observation of complications to enhance the therapeutic efficacy of surgery [13–15]. Targeted management is a high-quality management model developed in recent years and refers to the adoption of targeted perioperative management measures to promote early recovery and shorten the hospital stay of patients [16–18]. Fracture, surgery, and diabetes are prone to interact with each other and become a vicious circle. Perioperative targeted therapeutic interventions allow active control of blood glucose levels to closely observe the presence of diabetic complications. Psychological care improves patient compliance, and early functional exercise enhances patients' self-care ability, thereby promoting disease recovery and improving their quality of life. The greatest risks for patients with calcaneal fractures are nonhealing wounds, nonunion of the fracture and infection, so it is crucial to fully understand the condition of the diabetic patient and the medication used before surgery [19]. Diabetic patients with poor blood circulation in the heel require additional attention to blood circulation in the distal limb. Physical means and medications, including radiofrequency, laser, far infrared, and pneumatic pumps, are timely administered to protect the soft tissues and prevent local blister formation and skin breakdown to ensure a smooth procedure. Due to the paucity of clinical studies on the application of perioperative targeted management in patients with traumatic calcaneal fractures complicated by diabetes mellitus, this study aimed to investigate the effectiveness of the targeted management model on the rehabilitation process of patients with traumatic calcaneal fractures complicated by diabetes mellitus. The results of this study showed that the experimental group obtained a significantly shorter length of hospital stay and recovery time, and higher complete healing rates and Maryland scores versus the observation group, which was consistent with the research results by Wang Hongtao, suggesting that the targeted perioperative management effectively improves the fracture healing rate, reduces patients' pain, and improves patients' foot function after surgery. The reason may be that targeted treatment is tailored to the patient's specific situation and adjusted promptly according to their recovery. The psychological counseling of the patients before surgery significantly strengthens their treatment cooperation, and the close monitoring of the patient's vital signs and recovery after surgery allows for timely detection and management of abnormalities.

The article "The Efficacy of Targeted Perioperative Management for Diabetic Patients with Traumatic Calcaneal Fractures" was retracted in 2023. Reasons: unreliable results or conclusions; concerns about the data; concerns about the results or conclusions; concerns about the peer review.

Diabetes mellitus is associated with a slow recovery. A previous study indicated that patients with intraoperative hyperglycemia had higher anastomotic leakage rates than patients with a normal blood glucose level (12% versus 5%, *P* < 0.001) [19]. Therefore, a proper diet was necessitated to ensure enough nutrients for patients and enable better healing and faster recovery. The results of the present study showed that the experimental group showed better blood glucose results than the observation group, indicating the benefits of targeted perioperative management in the reduction and control of blood glucose. Moreover, the results of this study also revealed a higher safety profile of targeted perioperative management in comparison with conventional treatment, as evidenced by the lower incidence of complications in the experimental group versus the observation group, which may be attributable to the high quality of management that mitigated the surgical stress and enhanced the psychological status and prognosis of patients in the present study. The study by Zhang Lu et al. demonstrated that targeted management showed significant improvements in eliminating negative emotions, lowering the risk of complications, and relieving pain, which boosted postoperative recovery and ameliorated patients' quality of life. Furthermore, patients receiving targeted management in the present study were more satisfied with the treatment, which indicates that the protocol is feasible [20–22].

The article "The Efficacy of Targeted Perioperative Management for Diabetic Patients with Traumatic Calcaneal Fractures" was retracted in 2023. Reasons: unreliable results or conclusions; concerns about the data; concerns about the results or conclusions; concerns about the peer review.

To sum up, the application of targeted treatment in the perioperative management of diabetic patients with traumatic calcaneal fractures significantly promotes the recovery of patients, reduces the incidence of complications, increases treatment satisfaction, and ameliorates the doctor-patient relationship.

## Figures and Tables

**Figure 1:** Comparison of complete fracture healing rate. *Note*. *X*^2^ = 20.482, ^*∗∗∗*^*P* < 0.001 in the comparison of the number of completely healed cases between the two groups.

**Figure 2:** Comparison of Maryland scores (n (%)). *Note*. *X*^2^ = 22.844, ^*∗∗∗*^*P* < 0.001 in the comparison of the good rate of Maryland score between the two groups.

**Table 1:** Comparison of baseline features of the two groups (n (%)).

	Observation group (*n* = 50)	Experimental group (*n* = 50)	*t*/*X*^2^/*X*	*P*
*Gender*			1.644	0.841
Male	26	27		
Female	24	23		
Mean age	38.5 ± 4.2	38.3 ± 4.4	3.232	0.817

*Cause of injury*			1.674	0.457
Traffic accident	21	22		
Falling from height	17	16		
Sports injuries	12	12		

*Sanders fracture classification*			3.341	0.598
II	17	19		
III	21	20		
IV	12	11		

**Table 2:** Comparison of length of hospital stay and recovery time.

Groups	*n*	Length of hospital stay (d)	Recovery (d)	Duration of postoperative incisional oozing (d)
Observation group	50	15.28 ± 4.42	123.10 ± 22.82	5.71 ± 2.34
Experimental group	50	12.13 ± 3.77	111.22 ± 16.24	3.63 ± 1.04
*t*	—	3.834	2.999	5.744
*P*	—	<0.01	0.003	<0.01

**Table 3:** Comparison of complication rates.

	Observation group (*n* = 50)	Experimental group (*n* = 50)	*X* ^2^	*P*
Complication				
Incision infection	3	1	—	—
Delayed healing	1	0	—	—
Healing deformity	2	1	—	—
Joint pain	3	0	—	—
Complication rate (%)	9 (18)	2 (4)	5.005	0.025

**Table 4:** Comparison of treatment satisfaction.

	Observation group (*n* = 50)	Experimental group (*n* = 50)	*X* ^2^	*P*
Treatment satisfaction				
Satisfied	20	37	—	—
Basically satisfied	13	11	—	—
Dissatisfied	17	2	—	—
Total satisfaction rate (%)	33 (66)	48 (96)	14.62	<0.01

**Table 5:** Comparison of blood glucose ($\bar{x}\pm s$).

Groups	*n*	Fasting blood glucose (mmol/L)		Postprandial 2 h blood glucose (mmol/L)	
		Before treatment	After treatment	Before treatment	After treatment
Observation group	50	8.42 ± 1.22	7.96 ± 1.99	15.36 ± 2.42	14.22 ± 2.16
Experimental group	50	8.33 ± 1.13	7.01 ± 2.03	15.28 ± 2.35	12.38 ± 2.21
*t*	—	0.383	2.363	0.168	4.21
*P*	—	0.703	0.020	0.867	<0.001

The article "The Efficacy of Targeted Perioperative Management for Diabetic Patients with Traumatic Calcaneal Fractures" was retracted in 2023. Reasons: unreliable results or conclusions; concerns about the data; concerns about the results or conclusions; concerns about the peer review.

## Data Availability

The datasets used during the present study are available from the corresponding author upon reasonable request.

## References

[1] Dawson K. G., Jin A., Summerskill M., Swann D. (2021). Mobile diabetes telemedicine clinics for aboriginal first nation people with reported diabetes in British columbia. *Canadian Journal of Diabetes*.

[2] De Vries F., Lobatto D. J., Verstegen M. J. T., Van Furth W. R., Pereira A. M., Biermasz N. R. (2021). Postoperative diabetes insipidus: how to define and grade this complication?. *Pituitary*.

[3] Forde R., Arente L., Ausili D. (2021). The impact of the COVID-19 pandemic on people with diabetes and diabetes services: a pan-european survey of diabetes specialist nurses undertaken by the foundation of european nurses in diabetes survey consortium. *Diabetic Medicine: A Journal of the British Diabetic Association*.

[4] Liu Z., Yang L., Ding L., Wang L. (2021). Perioperative nursing care of vascular decompression for trigeminal neuralgia under AR medical technology. *Journal of Healthcare Engineering*.

[5] Manz J., Williams K., Jessen J., Kirkpatrick A. (2021). Addressing the perioperative nursing shortage via a perioperative nursing preceptorship for baccalaureate nursing students. *AORN Journal*.

[6] Marsh V., Kalisch B., McLaughlin M., Nguyen L. (2020). Nurses’ perceptions of the extent and type of missed perioperative nursing care. *AORN Journal*.

[7] Morawik I., Gospodarek M., Turżańska K., Zarębska A., Serefko A., Jabłoński M. (2020). The role of the perioperative nursing care in the satisfaction of patients after large joint replacements. *Wiadomosci Lekarskie*.

[8] Deleu P.-A., Leemrijse T., Chèze L. (2021). Post-sprain versus post-fracture post-traumatic ankle osteoarthritis: impact on foot and ankle kinematics and kinetics. *Gait and Posture*.

[9] Hosny H., Salama W., Marzouk A., Kenawey M. (2020). Repair of traumatic avulsed achilles tendon using double cerclage trans-calcaneal stainless steel sutures: prospective study and review of literature. *Injury*.

[10] Lê H. H., Lengelé J. P., Henin M., Toffoli S., Mineur P. (2021). Diabetes insipidus and acute myeloid leukemia harboring monosomy 7: report of two cases and literature review. *Acta Clinica Belgica*.

[11] Park E. S., Choi Y., Lee J., Park S.-H., Lee H. S. (2021). Calcaneal fracture: results of earlier rehabilitation after open reduction and internal fixation. *Archives of Orthopaedic and Trauma Surgery*.

[12] Rao K., Dibbern K., Day M., Glass N., Marsh J. L., Anderson D. D. (2019). Correlation of fracture energy with sanders classification and post-traumatic osteoarthritis after displaced intra-articular calcaneus fractures. *Journal of Orthopaedic Trauma*.

The article "The Efficacy of Targeted Perioperative Management for Diabetic Patients with Traumatic Calcaneal Fractures" was retracted in 2023. Reasons: unreliable results or conclusions; concerns about the data; concerns about the results or conclusions; concerns about the peer review.

[13] Polk C., Sampson M. M., Roshdy D., Davidson L. E. (2021). Skin and soft tissue infections in patients with diabetes mellitus. *Infectious Disease Clinics of North America*.

[14] Robertson G. L. (2021). Differential diagnosis of familial diabetes insipidus. *The Human Hypothalamus—Neuroendocrine Disorders*.

[15] Ueki K., Sasako T., Okazaki Y. (2021). Multifactorial intervention has a significant effect on diabetic kidney disease in patients with type 2 diabetes. *Kidney International*.

[16] Anaba P., Anaba E. A., Abuosi A. A. (2020). Patient satisfaction with perioperative nursing care in a tertiary hospital in Ghana. *International Journal of Health Care Quality Assurance*.

[17] Li L., Zhou J., Luo L., Chen X., Li Y. (2021). Application of the care bundle in perioperative nursing care of the type A aortic dissection. *International Journal of General Medicine*.

[18] Liu X.-Y., Jiao C.-H., Zhao D., Chen Y., Zhang H.-M. (2020). Psychological impact of high-quality nursing care on patients with esophageal cancer during perioperative period. *Medicine*.

[19] Reudink M., Huisman D. E., Van Rooijen S. J. (2021). Association between intraoperative blood glucose and anastomotic leakage in colorectal surgery. *Journal of Gastrointestinal Surgery*.

[20] Skou S. T., Juhl C. B., Hare K. B., Lohmander L. S., Roos E. M. (2020). Surgical or non-surgical treatment of traumatic skeletal fractures in adults: systematic review and meta-analysis of benefits and harms. *Systematic Reviews*.

[21] Wang B., Zhang X., Huo Y., Liu W., Wang W., Shao X. (2019). Calcaneal lengthening for partial traumatic loss of the calcaneus. *Injury*.

[22] Zhang L., Chen Y., Wang X. (2021). Simultaneous treatment of traumatic calcaneal osteomyelitis and defect deformity with near-arc bone transport by ilizarov technique. *Zhongguo Xiu Fu Chong Jian Wai Ke Za Zhi*.

